# *In Vivo* Growth Inhibition of Human Caucasian Prostate Adenocarcinoma in Nude Mice Induced by Amygdalin with Metabolic Enzyme Combinations

This article has been retracted.

**DOI:** 10.1155/2022/4767621

**Published:** 2022-05-21

**Authors:** Ahmed Mohammed Alwan, Jalil Tavakol Afshari

**Affiliations:** ^1^Department of Immunology and Allergy, Faculty of Medicine, Mashhad University of Medical Sciences, Mashhad, Iran; ^2^Section of Immunogenetic, Cell Culture Unit, Bu-Ali Research Institute, Mashhad University of Medical Sciences, Mashhad, Iran

## Abstract

Cancer of the prostate is an indicated type that is often recorded as a kind of cancer in men and the second critical cause of mortality through cancer cases. Many pharmacological investigations have shown that numerous herbal substances possess anticancer action. Amygdalin (AMD) has antitumour capabilities and works as an antioxidant, antibacterial, anti-inflammatory, and immune-regulating characteristics. The anticancer effects of amygdalin and its metabolizing enzymes, rhodanese (RHD) and betaglucosidase (BGD), were examined in vivo, as well as their antitumour processes. Novel, effective combination agents are necessary to increase existing cancer treatment rates. This research was aimed at determining the anticarcinogenic impact of amygdalin (AMD) in vivo. This research was aimed at determining the RHD and BGD on the anticarcinogenic impact of AMD in vivo. Subcutaneously, PC3 prostate cancer cell lines were implanted into nude mice. Mice were treated every day with 0.5 ml of 50 mg/ml (AMD), AMD+ (RHD 0.1 mg/ml), AMD+(BGD 0.1 mg/ml), and doxorubicin (DOX 50 mg/ml). Mice were normalized for negative control with untreated mice. In in vivo, morphopathological alterations in the tumour tissue were analyzed by histopathological staining methods. After 35 days of therapy, tumour growth and size inhibition were evident, indicating a function for the metabolic enzymes BGD and RHD in regulating AMD's anticancer effect in vivo. We concluded the critical role of metabolic enzymes BGD and RHD in elevating the antigrowth of PC3 cancer cell lines in Balb/c nude mice treated with AMD.

## 1. Introduction

Prostate cancer (PC) is by far the most widely recognized malignancy in males [1] and the second most common cancer mortality [2], with new cases expected to emerge globally and a high death rate [3]. Due to PC's great clinical and economic significance [4], extensive research has resulted in the fast growth of metastatic therapeutic options [5, 6]. AMD (Figure 1) (formerly known as laetrile) is a nitriloside present in the seed of prunasin group plants such as apricots, almonds, peaches, fruits, and many other rosaceous species [7, 8]. AMD has been commonly used to treat malignancy and pain [9–11]. AMD activation by BGD produces hydrocyanic acid, limiting cellular respiration and ultimately resulting in cell death. Cancer cells have a lower level of sulfur hydroxylase than healthy ones [9–13]. As a result, such cells can only detoxify the hydrocyanic acid produced during AMD hydrolysis. AMD's anticancer activity is enhanced when combined with BGD [10, 11, 13, 14]. In cancer cells, anaerobic glycolysis is the primary route [15]. Consequently, acidic circumstances boost betaglucosidase activity, which results in increased hydrocyanic acid and benzaldehyde formation and a deadly impact on cancer cells [12]. In contrast to other medications with low molecular weight, hydrocyanic acid is a nonspecific agent since it diffuses due to cyanide's toxicity and results in its removal. AMD concentrations less than 15 mmol/L were previously shown to be nontoxic to bladder cancer cells. However, activation of BGD reduced cell growth and migration [10, 14, 16]. Additionally, cells were arrested, and apoptosis was enhanced dose-dependently [17]. In recent years, the antitumour effect of AMD has been a gold stone topic [8, 9, 11]. It acts as an anticancer agent by liberating cyanogenic compounds in the body and leads to death of cancer cells, impeding tumour cell growth, and possibly reducing the occurrence of prostate cancer and some other types of cancer [17–19]. RHD is an enzyme of the normal cells that, in the presence of sulfur-containing chemicals, converts free cyanide to thiocyanate, a completely nontoxic molecule [20–22]. Thiocyanate is subsequently eliminated in the urine. RHD role can neutralize the AMD [19, 23–27]. As a result, these cells do not liberate HCN; from AMD, instead, it acts as glucose for healthy cells, supplying energy. In contrast, malignant cells lack RHD, and so the creation of HCN is stored in these cells [18, 28–30]. AMD may have a therapeutic impact on prostate cancer by inhibiting the viability of PC3 cells in vitro [17, 31, 32]. Additionally, no report of the same outcomes in vivo has been recorded. The indication of this research is to investigate the function of enzymatic control of AMD in vivo using BGD and RHD in nude mice tumoured with PC3 cell lines.

## 2. Materials and Methods

### 2.1. Animals

BALB/c (nude) mice (7 weeks of age, 24 ± 3.1 gram weight) were purchased from Iran's Pasteur Institute (NCBI) and housed for one week in the animal house of Mashhad University of Medical Sciences. Environment adaptation was used to normalize new settings for mice, which included in dividing the day into 2 halves, one of them dark and the other half is light, and a temperature of 22°C, with a portion of comprehensive food and water routine. Subcutaneous injection of PC3 cell lines was used to prepare mice for xenograft tumour induction. All conditions and handling with mice were included under class 2 biosafety cabinet. Food and water and all administrative solutions were sterilized carefully. All needs and conditions were met following animal rights and Mashhad University of Medical Sciences' guidelines for laboratory animals, which were approved using the ethical approval code [IR.MUMS.MEDICAL.REC.1397.417].

### 2.2. Chemical Reagents

AMD was obtained by Sigma-Aldrich Company (Germany, catalogue no. A6005), RHD was prepared by Sigma-Aldrich Company (Germany, catalogue no. G4511-5MG), BGD was brought from Sigma-Aldrich Company (Germany, catalogue no. R1756-5MG), and DOX was obtained by Merck Company (USA, CAS: 24385-10-2).

### 2.3. Cell Culture

Cell lines PC3 (human Caucasian prostate cancer) were acquired from Iran's Pasteur institution. RPMI culture medium (Gibco, Carlsbad, CA, USA) was used to culturing cells. Culture media were supplemented by FBS 10% and antibiotic 1% pen./strept. (Pan-Biotech, Germany). Cells were trypsinized with trypsin from Sigma-Aldrich Company (Germany) after culture and 75% growth (CAS: 9002-07-7) and cells were counted at a concentration of 106 cells/50 *μ*l PBS.

### 2.4. Tumour Induction

At a concentration of 2 × 10^7^ cells/50*μ*l PBS, cells were counted. Suspended cells were administered to each animal using insulin syringes. After seeing the first tumour bud (about ten days after cell injection), chemical compounds were delivered intraperitoneally into the treatment groups using an insulin syringe.

### 2.5. Treatment of Animals

Nude mice were divided into five groups and daily given 0.5 ml AMD alone, AMD 50 mg/ml+0.1 mg/ml RHD, or AMD 50 mg/ml+0.1 mg/ml BGD. Mice were administered with 1 *μ*M DOX doxorubicin as a positive control, whereas control animals were left untreated (002-07-7).

### 2.6. Tumour Volume Measurement

After visually inspecting and measuring the tumour with a calliper throughout the treatment procedure, the tumours were measured using a digital calliper every five days.

### 2.7. Animal Weight Measurement

For data analysis, the weights of all mice were determined every five days and compared to the untreated mice group.

### 2.8. Histopathology

Dissection of the mice resulted in the collection of representative tumours from each of the five groups in 10% neutral buffered formalin. The tumours were fixed in paraffin blocks, and standard Hematoxylin-Eosin staining was used to assess and compare histological features. Numerous characteristics such as tumour growth, mitotic index, and angiogenesis were investigated and compared in each animal group.

### 2.9. Data Analysis

The findings were provided as mean records and standard deviation. The data analyses were informed by using GraphPad Prism version 9.00, with significant differences proposed as *P* < 0.05.

## 3. Results

### 3.1. Tumour Volume

The volume of tumours in all mice groups did not record any change from day zero to the day 10. Tumours after day 10 started in the growth rates, and in untreated mice, continued in growth from day 10 to day 35. Tumours in mice treated with AMD+BGD was significantly inhibited, while they did not record significant inhibition in groups DOX and AMD+RHD (Figure 2).

### 3.2. Mouse Body Weight

The weight of mice did not show significant alterations in all groups (Figure 3).

### 3.3. Histopathological Analysis

Tumours from each of the five groups were collected and analyzed according to conventional histopathology procedures. Several microscopic aspects such as angiogenesis, invasiveness, and mitotic index were examined on Hematoxylin-Eosin-stained tumour sections. Angiogenesis was found in tumour sections from the control mice and mice treated with AMD, AMD+RHD, and AMD+BGD. Microscopic analysis of tumour sections demonstrated significantly more tumour growth and invasion in the control group than in the AMD, AMD+RHD, and AMD+BGD treatment groups. Treatment with AMD+BGD had a substantial effect on tumour growth morbidity compared to the other groups (Figure 4).

## 4. Discussion

The first objectives of this research was to verify the concept that amygdalin triggers growth inhibition in human prostate cancer cell line PC3 cells in vivo and to analyze its metabolic enzymes rhodanese and betaglucosidase as a potential adjunct to the existing prostate cancer therapy regimen (Figure 5). In in vivo, amygdalin injection reduced tumour development in PC3 cells through an apoptotic mechanism induced by betaglucosidase activation [32, 33]. According to specific research, cancer cells have a high concentration of betaglucosidase, which may be used to break down amygdalin and produce cyanide, which is harmful to cancer cells. According to several other research, rhodanese, which is capable of detoxifying cyanide, is secreted in normal cells but insufficient in malignant tumours [23, 34, 35]. The combination activity of the both of rhodanese and betaglucosidase may be the reason for producing cyanide in cancer cells treated with amygdalin which can be toxic for cancer cells while leaving normal cells unaffected [36, 37].

Further research is necessary to discover if betaglucosidase is concentrated in PC3 cells and rhodanese is absent and whether these characteristics are responsible for amygdalin's specificity for PC3 cell growth. Amygdalin was shown in this research to be capable of suppressing the progression of PC3 cell tumours in mice [17, 31, 38, 39]. As a result, we suspect that amygdalin decreases the viability of PC3 cells through a mechanism involving the betaglucosidase enzyme [17, 40]. Amygdalin substantially decreased the development of transplanted PC3 cell athymic mice through induction of the betaglucosidase enzyme, as reported in this work [41, 42]. The findings of our in vivo investigation are reporting nonpublished before. There were no apparent adverse effects seen in naked mice after amygdalin treatment. Amygdalin may be accurate since it naturally occurs as a plant or vitamin [43, 44]. Although it includes a harmful hydrocyanic group to live cells, it is harmless as long as the amygdalin component remains intact and does not release the hydrocyanic group enzymatically [11, 45].

## 5. Conclusion

Our study determined the inhibitory role of amygdalin treatment of PC3 in the mouse in vivo experiment. The mechanism of betaglucosidase and rhodanese played a critical role in controlling the efficacy of amygdalin. We suggested using amygdalin in more in vivo investigations to develop the treatment of cancer by cyanogenic glucoside compound.

## Figures and Tables

**Figure 1:** AMD structure.

**Figure 2:** Tumour volume analysis. (a) Graph of tumour volume analysis from day zero to day 35. (b) Comparison between groups one-way ANOVA *P* value < 0.05.

**Figure 3:** Mouse weight every five days during treatment.

**Figure 4:** Tumour histopathology. (a) Negative control group (untreated mice). (b) Mice treated with AMD+RHD. (c) Mice treated with AMD only. (d) Mice treated with DOX. (e) Mice treated with AMD+BGD.

**Figure 5:** RHD and BGD in controlling AMD in cancer and normal cells.

## Data Availability

All data are available within the manuscript, and additional data will be provided on request.
